# Characterization of an androgen-responsive, ornithine decarboxylase-related protein in mouse kidney

**DOI:** 10.1042/BSR20170163

**Published:** 2017-07-12

**Authors:** Kristian M. Silander, Päivi Pihlajamaa, Biswajyoti Sahu, Olli A. Jänne, Leif C. Andersson

**Affiliations:** 1 Department of Pathology, Haartman Institute, University of Helsinki, Helsinki, Finland; 2 Genome-Scale Biology Program, Research Programs Unit, Biomedicum Helsinki, University of Helsinki, Helsinki, Finland; 3 Institute of Biomedicine/Physiology, Biomedicum Helsinki, University of Helsinki, Helsinki, Finland

**Keywords:** androgen responsive, homo-dimer, ornithine decarboxylase, polyamines, ubiquitins

## Abstract

We have investigated and characterized a novel ornithine decarboxylase (ODC) related protein (ODCrp) also annotated as gm853. ODCrp shows 41% amino acid sequence identity with ODC and 38% with ODC antizyme inhibitor 1 (AZIN1). The *Odcrp* gene is selectively expressed in the epithelium of proximal tubuli of mouse kidney with higher expression in males than in females. Like *Odc* in mouse kidney, *Odcrp* is also androgen responsive with androgen receptor (AR)-binding loci within its regulatory region. ODCrp forms homodimers but does not heterodimerize with ODC. Although ODCrp contains 20 amino acid residues known to be necessary for the catalytic activity of ODC, no decarboxylase activity could be found with ornithine, lysine or arginine as substrates. ODCrp does not function as an AZIN, as it neither binds ODC antizyme 1 (OAZ1) nor prevents OAZ-mediated inactivation and degradation of ODC. ODCrp itself is degraded via ubiquination and mutation of Cys^363^ (corresponding to Cys^360^ of ODC) appears to destabilize the protein. Evidence for a function of ODCrp was found in ODC assays on lysates from transfected Cos-7 cells where ODCrp repressed the activity of endogenous ODC while Cys^363^Ala mutated ODCrp increased the enzymatic activity of endogenous ODC.

## Introduction

Polyamines are small ubiquitous aliphatic polycations involved in or are essential for fundamental cellular processes and events ranging from cell growth and proliferation to synthesis, function, and stability of macromolecules. Elevated polyamine levels have been linked to tumorigenesis. Thus, the intracellular polyamine concentration is tightly regulated at the levels of synthesis, catabolism, uptake, and excretion. Ornithine decarboxylase (ODC, EC 1.1.1.17) is the first and rate-limiting enzyme in the polyamine synthesis pathway [1–3].

The cellular ODC activity is regulated by a number of growth- and differentiation-inducing stimuli. ODC activity is tightly controlled by changes in the amount of catalytically active ODC protein [4,5]. ODC is catalytically active as a homodimer [6] with the monomers assembled in an antiparallel orientation [7,8]. As the monomers are rapidly dissociating and reassociating [9], ODC is inactivated and degraded by the polyamine-inducible protein ODC antizyme (OAZ) [10–12], which binds ODC monomers and targets them to ubiquitin-independent degradation by 26S proteasome [13–17]. Antizyme inhibitors (AZINs) are ODC-homologous proteins lacking catalytic activity [18]. AZINs, which bind OAZ with a higher affinity than ODC, sequester OAZ, and displace ODC from the ODC–OAZ complex enabling the formation of catalytically active enzyme [19,20]. AZINs that are often induced under same conditions as ODC [21] and are degraded by conventional ubiquitination [22,23].

The mouse protein ODCrp (ODC-related protein, also known as gm853 or ODC2/AZID) was first noticed in a phylogenetic analysis of 229 eukaryotic ODC/AZIN homologs, where the possible functions of the homologs were evaluated based on the conservation of 18 of the 20 amino acid residues found to be critical for the enzymatic ODC activity [24]. Homologs with conserved residues were viewed as potential catalytically active proteins. It was also suggested that homologs may function as antizyme inhibitors or form heterodimers with ODC [24] to inactivate, enhance, or protect the ODC in the complex. In the present study, we characterized the role and functions of ODCrp by investigating its expression profile, protein interactions, and enzymatic activity in the context of the known ODC-OAZ-AZIN regulatory system and possible formation of heterodimer with ODC. ODCrp contains a unique N-terminal extension of 14 amino acids, the possible role of which we also investigated.

## Materials and methods

### Materials

ODCrp cDNA (F520013M09, gm853) was purchased from ImaGenes (Berlin, Germany). The cDNA was subcloned into mammalian expression vectors pCDNA3.1 (Invitrogen, Thermo Fisher Scientific Inc., Waltham, U.S.A.), p3XFLAG-CMV-10, p3XFLAG-CMV-14 (Sigma–Aldrich, St. Louis, Missouri, U.S.A.) and a pCI-neo vector (Promega, Madison, Wisconsin, U.S.A.) modified to produce a C-terminal c-Myc tag. ODCrp cDNA was also modified; the first 13 residues were truncated (_Δ1–13_ODCrp) and/or Cys^363^ was mutated to alanine (_Δ1–13_ODCrp_C363A_ and ODCrp_C363A_). Primers used for cloning and qPCR were purchased from Oligomer Oy (Helsinki, Finland) or IDT (Integrated DNA Technologies, Coralville, Iowa, U.S.A.). The cloned constructs were verified by sequencing.

Two custom-made ODCrp antibodies were used. Rabbit anti-ODCrp[A] antibody, made by Agrisera (Vännäs, Sweden), was raised against the first 25 N-terminal residues of the protein (MNTPSEVKKDLLGVAEHLRPSEPIT). Rabbit anti-ODCrp[B] antibody, made by GenicBio (Shanghai, China), was raised against residues 305–318 (KKSSLDPGGHRKLA). The anti-ODCrp[A] antibody was used in immunohistochemistry and the anti-ODCrp[B] antibody, which also detects the N-terminally truncated form _Δ1–13_ODCrp, used in immunoblotting. All animals were handled in strict accordance with good animal practices as defined by the relevant Finnish animal welfare bodies, and the European Communities Council directive (86/609/EEC). The specificities of both antibodies were verified by SDS/PAGE and immunoblotting, and no cross-reactivity with ODC, AZIN1, or antizyme inhibitor 2 (AZIN2) was observed.

### Experimental animals

ICR mice (10- to 12-weeks old) were used. Intact males, orchiectomized males, and female mice were injected subcutaneously with testosterone (T, 1 mg/mouse/day in 0.1 ml mineral oil) or vehicle. Orchiectomized males received T four days after the operation. Gene expression analyses were performed with mice treated with T for 3 days. ChIP assays were performed 2 h after a single T injection. All animal experiments were approved by Finnish Review Board for Animal Experiments and performed according to the guidelines for animal experiments at the University of Helsinki (permit number ESLH-2008-09035/Ym23). The mice were killed by carbon dioxide inhalation and different organs were either snap-frozen in liquid nitrogen for RNA isolation or fixed in 10% buffered formalin (Sigma–Aldrich) and embedded in paraffin for immunohistochemistry.

### ChIP and ChIP-sequencing

Minced fresh mouse tissues were cross-linked in 1% formaldehyde (Merck KGaA, Darmstadt, Germany) at room temperature for 20 min. After washing twice with ice-cold PBS, tissues were homogenized in hexylene glycol buffer to isolate a crude nuclear fraction [25]. Sonication (Sonicator 3000, Misonix, Inc., Farmingdale, U.S.A.) was performed in 500 µl of RIPA buffer to yield chromatin fragments of 100–500 bp in size. Immunoprecipitation was carried out with polyclonal anti-androgen receptor (AR) antibody or normal rabbit IgG (sc-2027, Santa Cruz, Dallas, U.S.A.) as previously described [26]. After reverse cross-linking overnight at 65°C, immunoprecipitated and input DNA was purified using PCR purification kit (Qiagen, Hilden, Germany) and eluted in 100 µl of elution buffer. For ChIP qPCR, 5 µl of ChIP or input DNA was used in each reaction with SYBR Green master mix (Roche, Basel, Switzerland) and specific primers (*Odcrp* −4 kb: forward primer 5′-AGGGTCAGGATGTTCCTGTG, reverse primer 5′-GAGAGCTTTGGCTCCTGATG; *Odcrp* +30 kb: forward primer 5′-CAGCCCAGATGCAGAGTTTC, reverse primer 5′-TTCCAGCCTTTGAGTTTGCT). Results from IP samples were normalized to respective input sample, and the results (mean + S.E.M.) for four replicates are shown as percent of input. DNA libraries from ChIP samples were prepared according to Illumina’s instructions and sequenced using Illumina Genome Analyzer II. Peak calling was performed using MACS algorithm [27] and sequencing tag pile-up was visualized using Integrative Genomics Viewer [28].

### qPCR

Snap-frozen mouse organs (kidney, liver, brain, lung, spleen, heart, prostate, and testis) were powderized and RNA was isolated using TRI Reagent (RNA/DNA/Protein isolation reagent, Molecular Research Center Inc., Ohio, U.S.A.) according to the manufacturer’s instructions. RNA (1 µg) was used to produce cDNA (High Capacity RNA-to-cDNA Kit, Applied Biosystems, Life Technologies, Thermo Fisher Scientific Inc.) according to manufacturer’s instructions. The cDNA was then used as template in qPCR (LightCycler, Roche) with enzyme mix (SYBR Green/ROX qPCR Master Mix (2×), Thermo Scientific, Thermo Fisher Scientific Inc.) and specific primers (ODCrp: forward primer 5′-ACACACCTGAGAGCTACAGA and reverse primer 5′-TCCTGGATCTAGGGAAGACT, β2M: forward primer 5′-ATGTCTCGATCCCAGTAGAC and reverse primer 5′-GCTATCCAGAAAACCCCTCA). Sample quantitations were normalized using the invariant endogenous control β2M. Finally, the results (mean + S.D.) of three biological replicates were scaled to the result of untreated male control.

### Immunohistochemistry

Five-micrometer thick sections from formalin fixed and paraffin-embedded kidneys were stained with 1:1200 diluted rabbit anti-ODCrp[A] antibody and with its preimmune serum as control using Vectastain Elite ABC Kit (Vector Laboratories Inc., Burlingame, U.S.A.) according to the manufacturer’s instructions essentially as described [29]. Light microscope photographs were taken with an Olympus BX51 microscope (Olympus Optical, Tokyo, Japan) and a Nikon Digital Sight DS-5M camera (Nikon Corporation, Tokyo, Japan) using NIS-Elements F2.30 software (Nikon Corporation). Digital image processing was performed with PhotoScape v3.6.1 (Mooii Tech, Informer Technologies Inc., Los Angeles, U.S.A.).

### Cell cultures and transfections

Cos-7 cells were cultured in DMEM medium. ODC-deficient CHO cells (a kind gift from Dr Lo Persson, Lund, Sweden), devoid of endogenous ODC activity, were cultured in RPMI-1640 medium supplemented with putrescine. Both media also contained 10% (v/v) FBS (Gibco, Life Technologies, Thermo Fisher Scientific Inc.), L-glutamine and penicillin and streptomycin. ODC-deficient CHO cells were plated without putrescine 24 h before transfection. Cells were transfected with the desired plasmids using the FuGENE6 transfection reagent (Promega) according to the manufacturer’s instructions. In co-transfection experiments, the transfection mix contained equal amounts of both plasmids. Production of the transfected proteins was verified by SDS/PAGE and immunoblotting.

### *In-vitro* translation

Radiolabeled *in vitro* translated proteins were produced using an *In-vitro* translation (IVT) kit (TNT Coupled Reticulocyte Lysate System, Promega) according to the manufacturer’s instructions with L-[^35^S]-methionine (PerkinElmer, Waltham, U.S.A.). Samples of the translated proteins and Amersham Rainbow [^14^C] methylated protein molecular weight marker (Amersham Biosciences, GE Healthcare Life Sciences, Chicago, U.S.A.) were separated by SDS/PAGE (12% gel). The gel was fixed for 30 min in 30% methanol and 10% acetic acid solution and incubated for 1 h in Amplify Fluorographic Reagent (Amersham Biosciences). The gel was vacuum dried (Model 853 Gel Dryer, Bio–Rad, Hercules, U.S.A.) on to filter paper for 2 h at 80°C and used to expose an X-ray film (FUJI) overnight.

### Degradation assay

Protein degradation assay was performed as described previously [23]. Of the *in-vitro* translated proteins used, only ODC was radiolabeled. As a negative control, IVT lysate without translated proteins was mixed with radiolabeled ODC. The reactions were set up by mixing 1 µl OAZ with 14 µl ODCrp/_Δ1–13_ODCrp/AZIN1/lysate for 10 min at room temperature. ODC (2 µl) was added to the mixture, which was kept at 4°C for 5 min, whereafter prewarmed (37°C) ATP-regenerating buffer (50 mM Tris/HCl, pH 7.5, 5 mM MgCl_2_, 2 mM DTT, 0.5 mM ATP, 10 mM p-creatine, and 5 µg/ml creatine kinase) was added to a total volume of 60 µl. The reactions were incubated at 37°C and 5 µl samples were taken after 0, 10, 30 min, and 1 h. The samples were immediately mixed with 2× Laemmli sample buffer + 2-mercaptoethanol and separated by SDS/PAGE (12% gel). Radiolabeled ODC was visualized by fluorography.

### Catalytic activity assay

The decarboxylase activity assay was performed as described previously [23] by quantitating the release of ^14^CO_2_ from the radiolabeled substrates [1-^14^C]ornithine, [1-^14^C]arginine, or [1-^14^C]lysine (PerkinElmer). Reactions with *in-vitro* translated proteins contained 2 µl ODC, 1.4 µl OAZ, and 10 µl _Δ1–13_ODCrp/ODCrp/AZIN1 in different combinations. In the assays with cell lysates, Cos-7 or ODC-deficient CHO cells were transiently transfected with the empty pCDNA3.1 vector or constructs containing cDNA for ODC, AZIN1, ODCrp, _Δ1–13_ODCrp, ODCrp_C363A_, or _Δ1–13_ODCrp_C363A_. Transfected cells were collected and handled as described previously [30].

### Immunoprecipitation

In co-precipitation experiments, Cos-7 cells were co-transfected with plasmids producing FLAG-tagged and Myc-tagged proteins. Myc-tagged proteins were immunoprecipitated with 4 µg mouse monoclonal anti-Myc antibody (Sigma–Aldrich) and protein G-agarose (Roche) using an immunoprecipitation kit (Roche) according to the manufacturer’s instructions. Alternatively, FLAG-tagged proteins were immunoprecipitated with 4–5 µg mouse monoclonal anti-FLAG antibody (Sigma–Aldrich) and protein G-agarose. Finally, agarose pellets were suspended in 20 µl 2× Laemmli sample buffer + 2-mercaptoethanol, heated at 95°C for 5 min and separated by SDS/PAGE. Co-precipitated FLAG-tagged proteins were detected by immunoblotting with rabbit polyclonal anti-FLAG antibody (Sigma–Aldrich). Alternatively, co-precipitated Myc-tagged proteins were detected by immunoblotting with rabbit polyclonal anti-Myc antibody (MBL, Medical & Biological Laboratories Co., Ltd, Nagoya, Japan). In the ubiquitination experiments, Cos-7 cells were transfected with plasmids encoding FLAG-tagged proteins that were immunoprecipitated with mouse anti-FLAG antibody and analyzed by immunoblotting with rabbit anti-ubiquitin antibody (DAKO).

### Treatment with cycloheximide

Cos-7 cells were transfected with ODCrp-pCDNA3.1 or ODCrp_C363A_-pCDNA3.1 constructs and treated with 50 µg/ml cycloheximide. Samples were collected after 1, 3, and 5 h of treatment and lysed on ice in 60 µl cold Pawson lysis buffer for 10 min. Supernatants of centrifuged lysates were recovered for SDS/PAGE and analyzed by immunoblotting.

### Immunoblot analyses

Samples separated by SDS/PAGE were transferred to immunoblot membranes (Immobilon-FL transfer membranes, Merck Millipore, Darmstadt, Germany). After incubating the membranes with desired primary antibodies, the protein bands were visualized by incubating with appropriate fluorescent secondary antibodies; donkey anti-mouse (IRDye 800CW, Odyssey, LI-COR Biosciences, Lincoln, U.S.A.) and/or goat anti-rabbit (Alexa Flour 680, Invitrogen). All antibodies were diluted in 1:1 PBS + odyssey blocking buffer (LI-COR Biosciences). Finally, the membranes were scanned (Odyssey) and the images analyzed (ImageStudio Ver 3.1, LI-COR Biosciences).

### Statistical analysis

The statistical significance was calculated by unpaired Student’s *t* test, and a value of *P*<0.05 was considered significant. In the figures, the statistical significance of differences between two samples is indicated by a square bracket and an asterisk (*), except for Figure 7, which contains brackets only.

### Multiple sequence alignment

The multiple sequence alignment with mouse proteins ODCrp, ODC, AZIN1, and AZIN2 was performed with Clustal Omega 1.2.2 (ebi.ac.uk/Tools/msa/clustalo/). The GenBank IDs for the sequences used were AK143920.1, J03733.1, BC043722.1, and NM_172875.4, respectively. The sequence identities of the pairwise alignments were obtained using EMBOSS Needle (ebi.ac.uk/Tools/psa/emboss_needle/) with the default BLOSUM62 matrix.

## Results and discussion

### ODCrp and ODC/AZIN sequence alignment

The mouse ODCrp was first noticed in a phylogenic analysis of ODC-like sequences [24]. We aligned the sequences of mouse ODCrp, ODC, AZIN1, and AZIN2 in an attempt to uncover the function of ODCrp*.* As previously reported by Ivanov et al. [24], the following 20 amino acid residues are most critical for the catalytic ODC activity: Lys^69^ binds pyridoxal-5′-phosphate [31], residues Asp^88^, Glu^94^, Arg^154^, His^197^, Ser^200^, Gly^235–237^, Glu^274^, Arg^277^, Asp^332^, and Tyr^389^ stabilize the bound pyridoxal-5′-phosphate [7,8], residues Asp^332^ and Asp^361^ interact with the substrate [7,32], nucleophilic attack by Cys^360^ control the formation of the product [33], while Phe^397^ binds the L-CO_2_ [34]. Residues Gly^171^ and Gly^387^ have structural roles within the monomer [35], while residues Lys^169^, Arg^277^, Asp^332^, Asp^364^, and Tyr^389^ are important for the dimerization (Figure 1) [7,36]. Based on the conservation of the 20 functionally critical residues in ODCrp, Ivanov et al. [24] suggested that ODCrp might be catalytically active and able to form a dimer.

**Figure 1:** Multiple sequence alignment of the mouse ODCrp, ODC, AZIN1, and AZIN2 The 20 amino acid residues most critical for the catalytic ODC activity are marked in dark gray. The small arrow indicates the residue Cys^363^ in ODCrp and Cys^360^ in ODC. The antizyme-binding region is marked by a square. The five most important residues within the antizyme-binding region of ODC are marked in black, while the two residues of AZIN1 enhancing its affinity toward antizyme are marked in dark gray. Residues coming into close proximity with the surface of antizyme in the ODC-antizyme complex are marked in gray. Two of these residues also belong to the 20 most critical residues marked in dark gray, in that case, a gray dot (.) was placed above them. The two PEST sequences of ODC are marked with underlining bars, with the most important region marked in by a bolder bar. The alignment shows that ODCrp contains all the residues needed for catalytic activity, while the regions needed for antizyme binding and antizyme-mediated degradation are either mutated or missing. The alignment of the antizyme-binding regions of mouse and human ODC is also shown at the bottom. The two differing residues within the antizyme-binding region of mouse and human ODC are marked in gray.

OAZ binds to the 117–140 region of ODC [13]. The residues Gln^119^, Ala^124^, Asn^125^, Gln^129^, Glu^136^, Val^137^, and Met^140^ of human ODC are most important for OAZ binding [37]. Lys^141^ and Phe^397^ also interact with residues of OAZ, while Lys^69^, Lys^92^, and Tyr^323^ come in close proximity to the surface of OAZ [19]. Human and mouse ODC proteins differ at only two residues within the 117–140 region, where Asn^125^ and Val^137^ of human ODC are substituted for Ser^125^ and Ile^137^ in mouse ODC. In ODCrp, only 14 of the 24 residues of the OAZ-binding motifs are conserved, including only three (Ala^124^, Gln^129^, and Glu^136^) of the seven most important residues. However, of the other residues interacting with or coming in close proximity to OAZ, all except for Lys^92^ are conserved in ODCrp (Figure 1). AZINs have a higher affinity for OAZ than ODC [19]. The higher affinity is mediated by differences at residues 125 and 140, where serine and methionine of ODC are replaced by two lysine residues in AZIN1 [38]. In AZIN2, only the former lysine is conserved, while the latter is changed to alanine. It is unlikely that ODCrp has an AZIN-like affinity for OAZ, as in ODCrp these residues are arginine and isoleucine, respectively. ODC has two PEST sequences [39] that are recognized by the proteasome after OAZ binding to ODC [14]. The PEST sequences consist of regions 293–333 and 423–449, of which the latter is more important for the OAZ-mediated degradation [40]. In ODCrp, the region of the first PEST sequence has undergone many changes and is partially missing, while the latter region is lacking entirely (Figure 1). The mutated OAZ-binding motif suggests that ODCrp does not interact with OAZ, which together with the missing PEST sequences suggest that ODCrp degradation is likely to be initiated by ubiquitination.

The N- and C-terminal differences between ODCrp and ODC may not affect the functions of ODCrp, as those regions are located on the outer surface of the folded protein away from the active sites or dimer interface [41,8]. It is plausible to assume that ODCrp functions as an independent enzyme that does not interact with OAZ. Alternatively, ODCrp could serve as an ODC enhancer by binding ODC to form a catalytically active and/or a degradation-resistant heterodimers.

### Tissue expression and androgen responsiveness of Odcrp

According to the UniGene expressed sequence tag (EST) profile (Mm.387701) [42], *Odcrp* is mainly expressed in kidneys and to a lesser extent in liver. The result of qPCR experiments on RNAs from kidney, liver, brain, lung, spleen, heart, prostate, and testis showed that *Odcrp* mRNA is almost exclusively expressed in kidney, which is in-line with the EST profile. Although some expression was also found in the brain, the *Odcrp* mRNA level in the brain was only approximately 3% of that in the kidney. *Odcrp* mRNA level in the liver was less than 0.03% of that in the kidney (results not shown).

*Odc* is known to be androgen-inducible in mouse kidney [43–45]. qPCR experiments showed that the steady-state *Odcrp* mRNA level was approximately two-fold higher in male than in female kidneys. The difference in ODCrp expression in male and female kidneys was statistically significant (*P*<0.05) in a sample size of 17 male and 19 female mice. Treatment of ICR mice with 1 mg T for 3 days increased accumulation of *Odcrp* mRNA approximately 5.3-fold in male and 4.4-fold in female kidneys (Figure 2).

**Figure 2:** *Odcrp* mRNA is androgen responsive in mouse kidney Treatment of mice for 3 days with testosterone (+T, 1 mg/day) increased *Odcrp* mRNA accumulation by 5.3-fold in male and 4.4-fold in female kidneys as measured by qPCR. Results shown are the mean + S.D. of three replicates.

*In vivo* ChIP-seq experiments [46] were performed to examine whether there are AR-binding sites adjacent to the *Odcrp* locus to support the notion that androgen induction of *Odcrp* mRNA accumulation is a transcriptional event. AR binding *in vivo* to renal chromatin in the absence of androgen was marginal, while T treatment resulted in loading of AR on to specific sites adjacent to the *Odcrp* locus. More specifically, there were several AR binding events at +30 kb and −4 kb regions of the *Odcrp* transcription start site after 2 h of T exposure (Figure 3A). AR loading on to the two *Odcrp* regulatory regions was validated by using direct ChIP assays, and the results showed that androgen exposure result in approximately ten-fold enrichment of AR binding *in vivo* at both loci in murine kidneys (Figure 3B).

**Figure 3:** AR is loaded on to regulatory loci of *Odcrp* on mouse kidney chromatin AR loading *in vivo* was minimal in castrated male mice (Cast), and testosterone exposure induced approximately ten-fold enrichment of AR loading on to the −4 kb and +30 kb regulatory regions. Panel (**A**) shows the AR-binding events within and around the *Odcrp* locus as determined by ChIP-seq analysis. Panel (**B**) shows the results of direct ChIP assays on AR loading of four biological replicate samples normalized to the respective input samples (mean + S.E.M.).

Sections from kidneys of T treated and control male mice were stained with rabbit anti-ODCrp[A] antibody. In kidneys of control mice, ODCrp antigen level was most abundant in the subcapsular area and in the inner part of the cortex closest to the medulla, where the staining was strongest in the epithelial cells of the proximal tubules (Figure 4A). In kidneys of T-treated mice, ODCrp expression was seen throughout the whole cortex. Similar to ODC and AR expression [46,47], the staining of ODCrp antigen was strongest in the epithelial cells of the proximal tubules (Figure 4B). These cells also increased in size (Figure 4B), a known hypertrophic effect of androgens in mouse kidney [48]. Androgen regulation of *Odc* does not require catalytic ODC activity [44], and subsequent polyamine accumulation is not needed for androgen-induced hypertrophy of mouse kidney [44,49]. The effect of androgen action in mouse kidney comprises several hundreds of genes that are up- or down-regulated by androgens [46,50], and *Odcrp* belongs to the category of up-regulated genes. Of note, genes involved in DNA replication or cell proliferation are not regulated by androgens in mouse kidney as opposed to mouse prostate [46].

**Figure 4:** Immunohistochemically stained sections of mouse kidney All three panels (**A**,**B**,**C**) show a 50× magnified section of the whole cortex (**a**) as well as 200× magnified close ups of the subcapsular area (**b**) and inner cortex bordering the medulla (**c**). In normal male kidney (A), the presence of ODCrp antigen is confined to epithelial cells of the proximal tubules closest to the medulla and in the subcapsular area. Treating of male mice with T (1 mg/day) for 3 days (B) induced elevated ODCrp expression in the whole cortex, while still being most prominent in the proximal tubules of the inner cortex and subcapsular area. T also brought about hyperthrophy of proximal tubule epithelial cells. Panel (C) shows a kidney of T-treated male stained with preimmune serum. Nuclei were counterstained with hematoxylin.

### Catalytic activity and dimer formation of ODCrp

Dimerization is required for the catalytic ODC activity [6]. To investigate whether ODCrp is also capable of dimerization, Cos-7 cells were co-transfected with two ODCrp cDNA constructs, one producing a FLAG tag and the other a Myc tag. FLAG-tagged proteins were recovered by immunoprecipitation from cell lysates and analyzed by SDS/PAGE and immunoblotting with anti-Myc antibody. ODCrp was found to form dimers similar to ODC (Figure 5). In addition to native ODCrp, the modified forms _Δ1–13_ODCrp, ODCrp_C363A_, and _Δ1–13_ODCrp_C363A_ also dimerized. In _Δ1–13_ODCrp, the unique N-terminal extension was deleted while in ODCrp_C363A_, the Cys^363^ is mutated to alanine. Cys^363^ of ODCrp corresponds to Cys^360^ of ODC.

**Figure 5:** ODCrp dimers co-immunoprecipitated and visualized by immunoblotting Cos-7 cells were co-transfected with cDNAs encoding tagged proteins. The positive ODC-dimer control and two negative controls with only Myc-tagged ODCrp forms are on the left side of the markers (M). On the right side are the ODCrp samples with both FLAG- and Myc-tagged proteins. The FLAG-tagged proteins were immunoprecipitated with mouse anti-FLAG antibody, and co-precipitated Myc-tagged proteins were visualized by probing with rabbit anti-Myc antibody. The result shows that all four ODCrp variants formed homodimers.

We next investigated whether ODCrp catalyzes decarboxylation of ornithine. ODC-deficient CHO cells that are devoid of endogenous ODC activity [51] were transfected with cDNA constructs encoding different ODCrp variants or mouse ODC as positive control. Immunoblotting of the lysates from transfected cells showed protein expression with all cDNA constructs. However, in the ODC assay, only lysates from the cells transfected with ODC cDNA displayed catalytic activity above background (results shown in Supplementary Figure S1), which means that ODCrp itself does not display measurable decarboxylase activity under the conditions used for a conventional ODC assay.

Since ODCrp did not exert catalytic ODC activity, we tested whether ODCrp was able to catalyze decarboxylation of other substrates like lysine and arginine [52]. Constructs with different ODCrp cDNA variants were transfected into Cos-7 cells that are devoid of endogenous arginine and lysine decarboxylase activity. Lysates from transfected Cos-7 cells were assayed for lysine and arginine decarboxylase activity under the same conditions as that for the ODC assay. Since no positive controls were available for lysine and arginine decarboxylase assays, lysates of Cos-7 cells transfected with an ODC cDNA construct were assayed for ODC activity to serve as a positive control. No lysine or arginine decarboxylase activity was detected with the ODCrp constructs used, indicating that the substrate of ODCrp is neither lysine nor arginine (results shown in Supplementary Figures S2 and S3).

Ivanov et al. [24] originally suggested that ODCrp might form a heterodimer with ODC. To investigate this possibility, we co-transfected Cos-7 cells with cDNA constructs producing Myc-tagged (mouse) ODC and FLAG-tagged ODCrp proteins. As a positive control, Cos-7 cells were co-transfected with constructs producing Myc-tagged (mouse) ODC and FLAG-tagged (mouse) ODC. As a negative control, Cos-7 cells were co-transfected with Myc-tagged (mouse) ODC and FLAG-tagged (human) AZIN1. The Myc-tagged proteins were recovered by immunoprecipitation from lysates and analyzed by SDS/PAGE and immunoblotting with anti-FLAG antibody. Neither ODCrp nor _Δ1–13_ODCrp co-precipitated with ODC under the conditions where ODC-Myc co-precipitated with ODC-FLAG (Figure 6A). A reciprocal immunoprecipitation yielded the same result (shown in supplementary Figure S4 A,B). Thus, no evidence for formation of stable heterodimers between ODC and ODCrp was obtained.

**Figure 6:** ODC and OAZ co-immunoprecipitation and visualization by immunoblotting Cos-7 cells were transfected with cDNAs encoding tagged proteins. Panel (**A**) shows proteins immunoprecipitated with mouse anti-Myc antibody and immunoblotted with rabbit anti-FLAG antibody. The left side in panel (A) shows a negative control with only FLAG-tagged proteins. Although the negative controls should be clear, faint ODCrp and _Δ1–13_ODCrp bands can be seen due to unspecific binding. The fact that the bands are equally faint in the co-immunoprecipitation samples (right side in panel (A)) shows that ODCrp does not co-precipitate with ODC or OAZ, indicating that ODCrp does not form stable heterodimers. Panel (**B**) shows pre-immunoprecipitation samples probed with anti-FLAG (upper) and anti-Myc (lower) antibodies to verify the presence of transfected proteins. The samples in panel (B) are in the same order as in panel (A), except for the positive ODC – ODC control, which is replaced with marker.

Although ODCrp neither catalyzed ornithine decarboxylation nor formed dimer with ODC, it could nevertheless affect endogenous ODC activity by interacting with other endogenous proteins or by acting upon a substrate that is naturally present in the cells. To examine this possibility, we performed an ODC assay with lysates from Cos-7 cells transfected with cDNA constructs for the different ODCrp variants and with mouse ODC cDNA as positive control. Human AZIN1, which should bind the endogenous green monkey OAZ1 (human and green monkey OAZ1 are 99% identical), was also included to mark the highest activity achievable with endogenous ODC. Compared with the vector control, the presence of ODCrp and _Δ1–13_ODCrp had a weak but statistically significant repressing effect on the total ODC activity. This confirmed that ODCrp itself did not have any intrinsic ODC activity. On the contrary, expression of the mutated and ‘inactive’ counterparts ODCrp_C363A_ and _Δ1–13_ODCrp_C363A_ had a slight but statistically significant enhancing effect on the total ODC activity (Figure 7). The activities of the lysates with the different ODCrp forms were smaller than with AZIN1 and only approximately one-tenth of that with the positive control ODC (not shown), suggesting that the different ODCrp forms somehow affected the catalytic activity of endogenous ODC. The intact and mutated variants of ODCrp should essentially have the same molecular interactions, with the difference that the mutated forms should not catalyze decarboxylation [33]. If the concentration of this putative substrate is low and/or only a small fraction of it is free and metabolically available, as is the case with polyamines [53], and if both the intact and mutated ODCrp forms bind the substrate but only the intact forms complete the reaction, it could explain why the total ODC activity is repressed in the presence of ODCrp and _Δ1–13_ODCrp and increased in the presence of ODCrp_C363A_ and _Δ1–13_ODCrp_C363A_. These opposite effects seen with the intact and mutated forms are unlikely to result from differences in protein levels (further elaborated below) or cell proliferation, as immunoblotting revealed the presence of all ODCrp forms at similar total protein concentrations (shown in Supplementary Figure S5).

**Figure 7:** ODC assay on transfected Cos-7 cells Transfected Cos-7 cells were lysed directly in the assay buffer. The ODC activities of ODCrp, _Δ1–13_ODCrp, ODCrp_C363A_, _Δ1–13_ODCrp_C363A_, AZIN1, and vector control were all of the same order of magnitude. As compared with the vector control, the endogenous ODC activity was decreased by the presence of the ‘catalytically intact’ ODCrp forms and enhanced by the C363A mutated forms. Results are shown as the mean + S.D. of four replicates taken from separate cell culture dishes. All brackets indicate statistically significant differences.

### ODCrp degradation and stability

Unlike ODC, ODCrp is likely to be degraded by ubiquitination as both the OAZ-binding motifs and the two PEST sequences are impaired. To investigate the degradation pathway of ODCrp, FLAG-tagged proteins were recovered by immunoprecipitation from lysates of transfected Cos7-cells and analyzed by SDS/PAGE and immunoblotting with antiubiquitin antibody. ODCrp was found to be ubiquitinated like AZIN1 (Figure 8) [22]. No difference was observed between ODCrp and _Δ1–13_ODCrp.

**Figure 8:** Immunoprecipitated proteins blotted with antiubiquitin antibody FLAG-tagged proteins produced in Cos-7 cells were immunoprecipitated with mouse anti-FLAG antibody. The first four samples were immunoblotted with rabbit anti-ubiquitin antibody to show that ODCrp and _Δ1–13_ODCrp were ubiquitinated like the positive AZIN1 control, and the non-ubiquitinated ODC-FLAG served as negative control. The fifth sample is the ODC control reprobed with anti-FLAG antibody.

When verifying the amounts of transfected proteins in the ODC assay samples by SDS/PAGE and immunoblotting, we observed that the levels of ODCrp_C363A_ and _Δ1–13_ODCrp_C363A_ appeared lower than the levels of ODCrp and _Δ1–13_ODCrp. To examine the reason for this finding, cells transfected with ODCrp or ODCrp_C363A_ constructs were treated with 50 μg/ml cycloheximide, lysed, and the lysates were analyzed by immunoblotting with anti-ODCrp[B] antibody. The results showed that the mutation of Cys^363^ (corresponding to Cys^360^ of ODC) to alanine caused destabilization of ODCrp (Figure 9), suggesting that this residue is of importance for the functional role and/or conformation of the protein.

**Figure 9:** Stability of ODCrp as determined by cloheximide treatment Cos-7 cells transfected with ODCrp or ODCrp_C363A_ constructs were treated with cycloheximide (50 µg/ml) for 0, 1, 3, and 5 h. The relative amounts of ODCrp and ODCrp_C363A_ at different time points were quantitated in relation to respective GPADH bands on the immunoblot. The results are shown as the mean + S.D. of the band intensity of four sample replicates.

### Interaction between ODCrp and antizyme and the effect on ODC degradation

In ODC (and AZIN1), the residues 117–140 constitute the OAZ-binding motif [13]. Despite the fact that the sequence alignment showed that only 14 of these residues are conserved in ODCrp, an interaction between ODCrp and OAZ could still be mediated by residues outside of the OAZ-binding region. We performed a co-immunoprecipitation experiment to investigate whether ODCrp displays AZIN functions by binding to OAZ. Cos-7 cells were co-transfected with constructs producing FLAG-tagged ODCrp or AZIN1 and Myc-tagged OAZ. The Myc-tagged OAZ was recovered by immunoprecipitation from the lysates and analyzed by SDS/PAGE and immunoblotting with anti-FLAG antibody. There was no evidence for direct binding between ODCrp and OAZ, whereas AZIN1 co-precipitated with OAZ (Figure 6A, last two lanes).

The possibility exists that ODCrp inhibits the OAZ-mediated degradation of ODC without direct binding to OAZ. It is also possible that the interaction between ODCrp and OAZ or between ODCrp and ODC occurs even if it cannot be found by co-immunoprecipitation. To investigate this, we performed degradation assays with *in-vitro* translated proteins. The results showed that neither ODCrp nor _Δ1–13_ODCrp influences the OAZ-mediated degradation of ODC under the conditions where AZIN1 blocked ODC degradation (Figure 10). Thus, since ODCrp does not directly bind OAZ or protect ODC from OAZ-mediated degradation, it is very unlikely that ODCrp displays AZIN functions *in vivo*.

**Figure 10:** ODC degradation assay with *in vitro* translated proteins *In vitro* translated (IVT) proteins were mixed in a 2:1:14 ratio of ODC:OAZ1:ODCrp/_Δ1–13_ODCrp/AZIN1/lysate, respectively, where only ODC was radiolabeled. The reaction with only ODC and IVT lysate (devoid of translated proteins) shows the basal rate of ODC degradation. Adding OAZ1 (OAZ + IVT lysate) to the reaction increased the rate of degradation. ODCrp (OAZ + ODCrp) and _Δ1–13_ODCrp (OAZ + _Δ1–13_ODCrp) did not rescue ODC from the OAZ-mediated degradation, whereas ODC degradation was markedly slowed down in the presence of AZIN1 (OAZ + AZIN1).

To further investigate functional interactions between ODC, OAZ, ODCrp, and AZIN1, we performed ODC assays with *in-vitro* translated proteins. The results showed that: (i) ODCrp did not release ODC from OAZ-mediated inhibition under conditions where AZIN1 displayed such a function, and (ii) the activity of 10 µl IVT ODCrp was very close to that of 10 µl AZIN1 and less than approximately one-third of the activity of 2 µl ODC, suggesting that ODCrp was devoid of measurable intrinsic ODC activity under the conditions where the positive ODC control catalyzed ornithine decarboxylation as expected (Figure 11). We could not get evidence for any functional or regulatory role of the unique N-terminal extension ODCrp.

**Figure 11:** ODC activity assay with IVT proteins The assay sets contained 2 µl ODC, 1.4 µl OAZ, and 10 µl ODCrp/_Δ1–13_ODCrp/AZIN1 in different combinations. The activity of 10 µl ODCrp and _Δ1–13_ODCrp was similar to the activity of 10 µl AZIN1 and lower than that of 2 µl ODC, suggesting that ODCrp and _Δ1–13_ODCrp have no intrinsic ODC activity. Unlike AZIN1, ODCrp or _Δ1–13_ODCrp did not block the antizyme-mediated inhibition of ODC, as the measured activity of the reaction set containing all three components was essentially the same as the calculated additive activity of the two separate ‘basal’ reactions (as the values on the bars indicate). Thus, ODCrp is not an AZIN. Results are shown as the mean + S.D. of three to five reactions per set.

## Conclusion

ODCrp is an androgen-inducible protein specific to mouse kidney, where its expression is most prominent in epithelial cells of the proximal tubules closest to the medulla. ODCrp is neither an AZIN nor a direct ODC enhancer, as no interaction could be shown between ODCrp, and OAZ or ODC. While ODCrp forms dimers, it does not catalyze decarboxylation of ornithine, lysine, or arginine. Its putative substrate remains to be identified. However, ODCrp displayed a small but significant regulatory influence on the catalytic activity of endogenous ODC. Last, no indication for a functional or regulatory role of the unique N-terminal extension ODCrp was uncovered.

## Supporting information

**Supplementary Fig. S1:** ODC assay with transfected ODC-deficient CHO cells. Transfected ODC-deficient CHO cells were lysed directly in the assay buffer. These cells are devoid of endogenous active ODC. None of the ODCrp forms exhibited activities over the lysate control, whereas the activity of the positive ODC control was over 1000-times higher than the rest of the samples **(A)**. Thus, ODCrp does not catalyze decarboxylation of ornithine. Results are shown as the mean + SD of duplicate or triplicate replicates. The experiment was repeated three times with similar results. In panel **B** samples of lysates were probed with anti-ODCrp[B] and anti-GAPDH antibodies verifying the presence of the transfected proteins and equal loadings.

**Supplementary Fig. S2:** Lysine decarboxylase assay with transfected Cos7 cells. Transfected Cos7 cells were lysed directly in the assay buffer. None of the ODCrp forms exhibited activities over the lysate control **(A)**. ODCrp did not catalyze decarboxylation of lysine. Lysates of Cos7 cells transfected with ODC cDNA were assayed for ODC activity as a positive control for the experimental setup. Results are shown as the mean + SD of two replicates. In panel **B** samples of lysates were probed with anti-ODCrp[B] antibodies verifying the presence of the transfected proteins.

**Supplementary Fig. S3:** Arginine decarboxylase assay with transfected Cos7 cells. Transfected Cos7 cells were lysed directly in the assay buffer. None of the ODCrp forms exhibited activities over the lysate control **(A)**. ODCrp did not catalyze decarboxylation of arginine. Lysates of Cos7 cells transfected with ODC cDNA were assayed for ODC activity as a positive control for the experimental setup. Results are shown as the mean + SD of two replicates taken from separate cell culture dishes. The experiment was repeated two times with similar results. In panel **B** samples of lysates were probed with anti-ODCrp[B] and anti-GAPDH antibodies verifying the presence of the transfected proteins and equal loadings.

**Supplementary Fig. S4:** ODC and OAZ co-immunoprecipitation and visualization by immunoblotting. Panel A and B show reciprocal experiment of that represented in Fig. 6 in main text. Cos-7 cells were transfected with cDNAs encoding tagged proteins. To the right of the marker (M) are proteins immunoprecipitated with mouse anti-FLAG antibody and immunoblotted with rabbit anti-Myc antibody. Pre-immunoprecipitation samples are to the left of the marker. Pre-immunoprecipitation samples were immunoblotted with both anti-FLAG and anti-Myc antibodies to verify the presence of transfected proteins. In panel **A**, only ODC-FLAG co-precipitated with ODC-Myc, indicating that ODCrp and _Δ1–13_ODCrp do not form stable dimers with ODC. In panel **B**, only AZIN1-FLAG co-precipitated with OAZ-Myc, verifying that ODCrp and _Δ1–13_ODCrp do not form stable dimers with OAZ.

**Supplementary Fig. S5:** Lysate samples of transfected Cos7 cells used in ODC assay (related to Fig.7 of main text). Transfected Cos7 cells were lysed directly in the assay buffer. Every immunoblotted sample represents separate ODC assay samples taken from individual cell culture dishes. Immunoblotting with anti-ODCrp[B] antibody verified the presence of transfected proteins and anti-GAPDH antibody shows equal loadings.

**Supplementary Fig. S6:** Validation of anti-ODCrp antibody specificities. Lysates of Cos7 cells transfected with cDNA for FLAG tagged ODCrp, _Δ1–13_ODCrp, (mouse) ODC, (human) AZIN1 and (human) AZIN2 were immunoblotted with anti-ODCrp[A] antibody (**A**) and anti-ODCrp[B] antibody (**B**). Neither antibody show any cross-reactivity with ODC, AZIN1 or AZIN2. Re-probing with anti-FLAG antibody shows presence of all transfected proteins.

**Supplementary Fig. S7:** Predicted ODCrp protein model. The functional form of ODCrp may resemble the 3D model of an ODCrp homodimer predicted and generated by SWISS-MODEL based on the human ODC homodimer template. Panel **A** show the predicted 3D model of an ODCrp homodimer where the protein backbone is shown in ribbon form and the side chains of the 20 critical amino acid residues are shown as stick models. The two subunits are presented in different colors. Panel **B** show a close up of both active sites and panel **C** shows a close up of one active site with the pyridoxal-5′-phosphate-binding Lys81 (corresponding to Lys69 of ODC) and the nucleophile Cys363 (corresponding to Cys360 of ODC). The 3D model of ODCrp was generated by the fully automated protein structure homology-modeling server SWISS-MODEL (swissmodel.expasy.org)^1,2,3,4^. The template recognition and structure modeling algorithm identified human ODC (1d7k.1.B) as the model with highest quality among the template library (SMTL version 2016-10-12, PDB release 2016-10-7). ODCrp residues 26-422 were aligned and used to build the 3D model. The model was built as a homodimer according to matching predictions (ProMod3 Version 1.0.1.). The GMQE (Global Quality Estimation) for the model was 0.76. However, the composite scoring function for the estimation of the global and local model quality (QMEAN) for the model was only -1.31. The pictures of the 3D model were generated using PyMOL (The PyMOL Molecular Graphics System, Version 1.8 Schrödinger, LLC.). (1) Biasini M, Bienert S, Waterhouse A, Arnold K, Studer G, Schmidt T, et al. SWISS-MODEL: modelling protein tertiary and quaternary structure using evolutionary information. Nucleic Acids Res 2014 Jul;42(Web Server issue):W252-8. (2) Arnold K, Bordoli L, Kopp J, Schwede T. The SWISS-MODEL workspace: a web-based environment for protein structure homology modelling. Bioinformatics 2006 Jan 15;22(2):195-201. (3) Kiefer F, Arnold K, Kunzli M, Bordoli L, Schwede T. The SWISS-MODEL Repository and associated resources. Nucleic Acids Res 2009 Jan;37(Database issue):D387-92. (4) Guex N, Peitsch MC, Schwede T. Automated comparative protein structure modeling with SWISS-MODEL and Swiss-PdbViewer: a historical perspective. Electrophoresis 2009 Jun;30 Suppl 1:S162-73.

## Abbreviations

AR: androgen receptor
AZIN1: antizyme inhibitor 1
AZIN2: antizyme inhibitor 2
ChIP: chromatin immunoprecipitation
EST: expressed sequence tag
IVT: *in-vitro* translation
OAZ: ornithine decarboxylase antizyme
ODC: ornithine decarboxylase
ODCrp: ornithine decarboxylase-related protein
qPCR: quantitative polymerase chain reaction
T: testosterone
